This article has been retracted.

# OTUB2 Facilitates Tumorigenesis of Gastric Cancer Through Promoting KDM1A-Mediated Stem Cell-Like Properties

**DOI:** 10.3389/fonc.2021.711735

**Published:** 2021-09-27

**Authors:** Guangming Liu, Wei Guo, Junjie Qin, Zhiliang Lin

**Affiliations:** ^1^ Department of Gastroenterology, The First Hospital of Jilin University, Changchun, China; ^2^ Department of Hematology, The First Hospital of Jilin University, Changchun, China; ^3^ Department of Colorectal Disease Specialty, Intestinal Microenvironment Treatment Center of General Surgery, Shanghai Tenth People’s Hospital, Tenth People’s Hospital of Tongji University, Shanghai, China

**Keywords:** gastric cancer, OTUB2, KDM1A, cancer stem cells, OTUB2/KDM1A

## Abstract

Otubain 2 (OTUB2), a deubiquitinating enzyme, overexpression is considered to predict poor outcome in various cancers. However, the function and potential regulatory mechanisms of OTUB2 in gastric cancer (GC) progression remains unclear. To determine how OTUB2 participate in GC progression, the gain and loss of-function experiments were conducted *in vivo* and *in vitro*. We found that OTUB2 was upregulated in GC samples (n=140) and cells. Moreover, the overall, first progression and post progression survival rates of GC patients with high OTUB2 expression showed a poorer prognosis than that in those patients with low OTUB2 expression. Down-regulation of OTUB2 suppressed sphere formation and reduced expression of stem cell markers in GC cells. Furthermore, OTUB2-silenced GC cells also showed a decreased proliferation, invasion, migration, and *in vivo* tumorigenic ability. However, OTUB2 overexpression showed the opposite effects. Notably, we demonstrated that OTUB2 increased lysine-specific histone demethylase 1A (KDM1A) expression through deubiquitination. KDM1A, a demethylase known to promote demethylation of downstream genes, was identified to promote the maintenance of cancer stem cell characteristics. Moreover, the alterations caused by OTUB2 overexpression were partly inversed by KDM1A knockdown and in turn KDM1A overexpression reversed the changes induced by OTUB2 shRNA. Taken together, we demonstrate that OTUB2 may serve as a vital driver in GC tumorigenesis by enhancing KDM1A-mediated stem cell-like properties.

## Introduction

Gastric cancer (GC) is one of the deadliest cancers and the fifth most common cancer globally (1). Although in the past few decades, the global incidence of GC has decreased significantly and the long-term survival rate has increased, it still remains an important contributor to the global cancer burden (2). At present, surgical resection is considered as the only radical treatment. With the improvement of treatment methods, the 5-year survival rate of patients has been greatly improved (3). However, lymph node metastasis was occurred in nearly a quarter of patients after surgery, the five-year overall survival rate still remains unsatisfactory (4). Therefore, it is necessary to explore the pathogenesis and potential therapeutic targets of GC.

Otubain 2 (OTUB2) is a member of OTUs superfamily and is first discovered in ovarian tumor gene from Drosophila melanogaster (5). OTUB2 exerts multiple functions, including regulating cancer progression. OTUB2 often acts as a cancer-promoting factor in cancer progression. For instance, OTUB2 was overexpressed in non-small cell lung cancer (NSCLC) and promoted the development of NSCLC (6). Overexpression of OTUB2 was also observed in liver cancer tumor tissues and cell lines and acted as a positive indicator for the poor prognosis of liver cancer patients (7). OTUB2 inhibition suppressed the development of papillary thyroid carcinoma (8). Those findings highlight the importance of OTUB2 in cancer progression. However, the function of OTUB2 in GC is still unknown.

The ubiquitin-proteasome system serves as the main regulator of protein post-translational modification, mediated by E1, E2, and E3 ubiquitin ligases and deubiquitinating enzymes (9). OTUB2 is a deubiquitinating enzyme, which is considered to be a key regulator of cancer cell cycle and signaling pathways (10). Early studies have shown that OTUB2 increased the stability of U2AF2 through deubiquitination and further promoted the Warburg effect and tumorigenesis of NSCLC (6). Notably, OTUB2 is considered to affect the properties of cancer stem cell (CSC) by regulating the ubiquitination of downstream genes, such as YAP/TAZ (11). CSC is regarded as an important cause of cancer treatment burden (12). CSCs have many biological properties, including the self-renewal, high tumorigenesis and invasiveness, chemotherapeutic resistance, and recurrence (13, 14). Therefore, exploring suitable targets to regulate CSCs properties will bring new ideas to the treatment of GC. Based on the above, we speculated that OTUB2 might regulate the properties of GC stem cells through the deubiquitination of downstream genes.

The lysine-specific histone demethylase 1A (KDM1A/LSD1), the first demethylase to be discovered, demethylates both mono- and di-methylated lysine -4 and -9 of the histone H3 (15). KDM1A also demethylates non-histone substrates, including DNA methyltransferase 1 (DNMT1) (16), early 2 factor (E2F) (17), p53 (18), and signal transducer and activator of transcription 3 (STAT3) (19), those factors play a vital role in GC progression. Additionally, KDM1A inhibition was reported to suppress the malignant phenotype of GC cells (20, 21). Altogether, the findings demonstrate that KDM1A may be a potential target for GC treatment. UALCAN website (http://ualcan.path.uab.edu/index.html) analyzed that OTUB2 and KDM1A were highly expressed in GC tissues, and their expressions were significantly positively correlated (**Figure 1**). Furthermore, considering OTUB2 is a member of deubiquitinating enzymes (DUBs) family, we thus investigated OTUB2 whether regulated the ubiquitination of KDM1A in GC cells.

**Figure 1:** Otubain 2 (OTUB2) is highly expressed in gastric cancer (GC) tissues and OTUB2 overexpression is preferentially connected with poor prognosis of patients with GC. **(A)** The data of OTUB2 expression was extracted from The Cancer Genome Atlas (TCGA) database and analyzed by the UALCAN website. **(B, C)** The expression of OTUB2 in GC tissues and para-carcinoma tissues was measured by quantitative Real-Time PCR (n = 140) and immunohistochemical staining. **(D)** The ratio of high expression of OTUB2 to low expression of OTUB2 in cancer tissues and adjacent tissues. **(E)** Survival rate of patients with GC analyzed by Kaplan-Meier plotter database. Data was represented as mean ± SD. **P < 0.01, ***P < 0.001.

The current study is the first to explore the effect of OTUB2 on the characteristics of GC stem cells and its potential regulatory mechanism. Our study may offer the theoretical basis for the clinical treatment of GC patients.

## Methods

### Clinical Data and Cell Culture

All the 140 pairs of normal and GC tissues were obtained from The First Hospital of Jilin University. The GC specimens used in present study were confirmed as GC tissues by pathology before experiment. All the patients did not receive preoperative or postoperative non-drug therapy. The study were approved by the Ethics Committee of The First Hospital of Jilin University and performed in accordance to World Medical Association Declaration of Helsinki and obtained the informed consent from all patients.

Human GC cell lines (MKN-45, SGC-7901, SNU-1, HGC-27, and AGS) and gastric epithelial cells-1 (GES-1) cells were purchased from Procell Life Science&Technology Co,.Ltd (Wuhan, China). The cell lines were placed in incubator with 5% CO_2_ at 37°C in RPMI-1640 medium (Sigma-Aldrich, Saint Quentin Fallavier, France) or Dulbecco’s modified Eagle’s medium (DMEM, Procell) containing 10% fetal bovine serum (FBS, Beyotime Biotechnology, Shanghai, China).

### Cell Transfection

The shRNAs against OTUB2 were purchased from GeneChem Group (Shanghai, China). The pcDNA3.1 plasmids were obtained from AxyBio (Changsha, China). MKN-45 and SGC-7901 cells were transfected with pcDNA3.1-OTUB2 (OTUB2) or its negative control (NC). HGC-27 and AGS cells were transfected with shRNA-OTUB2 (shRNA1 and shRNA2) or shRNA-NC (shNC). The transfections were mediated by Lipofectamine^®^3000 (Thermo Fisher, Waltham, MA, USA).

### Quantitative Real-Time PCR (qRT-PCR)

Total RNA was obtained from GC tissues and cells using the Trizol reagent (Invitrogen, Carlsbad, CA, USA). The complementary DNA (cDNA) was converted by RNA with the help of RNase inhibitor (Tiangen, Beijing, China) and SuperScript II reverse transcriptase (Invitrogen). Then, qRT-PCR analysis was performed using Roche Light-Cycler system (Roche, Basel, Switzerland) with SYBR Green reaction mix (Qiagen, Hilden, Germany). The OTUB2 expression was standardized by β-actin expression. The 2^-△△ct^ comparative method was used to calculate the relative expression levels. The primers used for qRT-PCR were: (OTUB2) 5’-ACACTTGGAACCGGCTTGAC-3’ (F); 5’-AGCACACGGACTGTCCTGA-3’ (R). (β-actin) 5’-GTCATTCCAAATATGAGATGCGT-3’ (F); 5’-GCATTACATAATTTACACGAAAGCA-3’ (R).

### Immunohistochemical Staining

The tissues were sectioned and incubated in hydrogen peroxide (3%) for 20 min at room temperature to eliminate endogenous peroxidase activity. Thereafter, the slices were blocked with normal goat serum (Dako Corporation, Carpinteria, CA, USA) for 15 min and then treated with primary antibodies. The primary antibodies against OTUB2 (Affinity, Catalog No. AF9147; Affinity Biosciences, OH, USA), Ki67 (Abcam, Catalog No. ab15580; 1:100; Cambridge, MA, USA), and lysine-specific histone demethylase 1A (KDM1A; Affinity, Catalog No. DF6290) were treated overnight at 4°C. After washing with PBS, the sections were incubated with horseradish peroxidase (HRP)-labeled secondary antibodies (Proteintech, Catalog No. SA00001-2; Wuhan, China) at a dilution of 1:500 for 2 h at 37°C. After washing, staining was performed using DAB reagent and the slices were counterstained with hematoxylin. An olympus microscope (Tokyo, Japan) (magnification, ×200) was used to observe and obtain the staining images.

### Western Blot Analysis

Total protein samples were obtained from the GC tissues and cells using the Tissue Protein Extraction Reagent (Thermo Fisher). The bicinchoninic acid (BCA) Protein Assay Kit (Thermo Fisher) was used to detect the concentration of protein. After separated by SDS-PAGE gel lectrophoresis, the proteins were transferred to the PVDF membranes. After treating with 5% skimmed milk, the membranes were treated with the primary antibodies and then the HRP-labeled secondary antibodies (1:5000, Abcam). Finally, the proteins in the membranes were visualized by chemiluminescence reagent and the optical density (OD) values were analyzed. β-actin was used as internal control to standardize the protein expression. The antibodies used were follows: OTUB2 (Affinity, Catalog No. AF9147; 1:1000), KDM1A (Affinity, Catalog No. DF6290; 1:1000), Nang (Abcam, Catalog No. ab109250; 1:1000), ALDH (Abcam, Catalog No. ab134188; 1:500), Oct4 (Abcam, Catalog No. ab19857; 1:1000), and β-actin (Abcam, Catalog No. ab8226; 1:2000).

### Sphere-Formation Assays

The GC cells (2 × 10^3^ cells) were seeded into an ultra-low-attachment 6-well plate. The plate was then treated with serum-free DMEM/F12 medium (Invitrogen) containing B27 (2%, Gibco BRL, Grand Island, NY, USA), EGF (10 ng/ml, Gibco BRL), and bFGF (20 ng/ml, Gibco BRL). Replacing the medium every 5 days, after two weeks, the sphere number was calculated.

### Flow Cytometric Analysis of CD44 Positive Cells

The GC cells (Semi-confluent, 70-90%) in the culture dish were washed with PBS and then dissociated from the dish by 0.25% Trypsin-EDTA. After centrifugation, the cell pellets were resuspended and treated with Fluorescein isothiocyanate (FITC)-CD44 antibody (Abcam, Catalog No. ab30405) or Phycoerythrin (PE)-conjugated CD133 antibody (1:200;Abcam, Catalog No. ab253271) on ice for 30 min. After washing with PBS, a BD FACSC alibur flow cytometer (Catalog No. 342976, BD Biosciences, San Jose, CA) was used to sort the CD44/CD133-positive cells.

### MTT Assay

GC cells (2 × 10^3^ cells/well) in logarithmic growth phase were seeded into 96-well plates. MTT solution (20 μl) was added into the plates on days 1, 2, and 3. After incubated in an incubator for 4 h at 37°C, cells were treated with DMSO. After 10 min in the dark, the absorbance values of 570 nm were detected by a microplate reader (Biotek, Winooski, VT, USA).

### 5-Ethynyl-2-Deoxyuridine (EdU) Assay

The GC cell proliferation was assessed using an EdU assay kit (RiboBio, Guangzhou, China). Briefly, GC cells (1 × 10^4^ cells) were seeded into the 96-well plate and incubated in an incubator at 37°C overnight. Afterwards, the EdU solution (25 μM) was added to the 96-well plate for 24 h and then cells were permeabilized for 10 min by using 0.5% TritonX-100. After treated with Apollo reaction solution (200 μl) for 30 min, cells were treated with DAPI to stain the nuclei. Finally, a fluorescence microscope (Olympus, 400 ×) was used to observe cell proliferation.

### Wound Healing Assay

Wound healing assay was conducted to assess the cell migration capacity of GC cells. In brief, cells were seeded into the 12-well plates. After grew to confluence, cells were wounded by scraping with a pipette tip (200 μl). Afterwards, cells were washed with serum-free medium and placed into the regular medium. Finally, wounds were observed at 0, 24, and 48 h, and the migration distance was calculated.

### Transwell Assay

The transwell chamber (Corning Life Sciences, Bedford, MA, USA) with Matrigel gel−coated membranes was placed in 24-well plates. The lower chamber was added with 800 μl culture solution containing 30% FBS. The upper chamber was added with 200 μl cell suspension at a density of 1×10^4^ cells/well. After incubation in a cell culture incubator at 37°C supplied with 5% CO_2_ for 24 h, the Transwell chamber was washed with PBS to remove non-invaded cells. Then the cells on the lower chamber were fixed with paraformaldehyde (4%) at room temperature for 25 min and then stained with crystal violet solution (0.4%) for 5 min. Cells on lower chamber were counted under an Olympus microscope (×200). Five fields were selected for each sample, and mean values of cell numbers were counted.

### *In Vivo* Tumor Formation

All the animal experiments were performed according to the National Institutes of Health guide for the care and use of Laboratory animals and laboratory safety and biosecurity (22, 23). Male BALB/c nude mice (6 weeks) were obtained from Slac Laboratory Animal Center (Shanghai, China). Stable OTUB2 overexpression (SGC-7901 cells, 4 × 10^5^ cells) or low expression (HGC-27, 4 × 10^5^ cells) cells were subcutaneously injected into the mice. The tumor size was detected every 5 days. After 35 days, all nude mice were euthanized and tumor weight was recorded. The animal experiments were conducted by the approval of The First Hospital of Jilin University and in accordance to the Guide for the Care and Use of Laboratory Animals.

### Co-Immunoprecipitation Detection and Deubiquitination Assay

Cells were incubated in lysis buffer containing protease inhibitor Cocktail (Roche, Mennheim, Germany) for subsequent co-IP. The cell lysates were incubated with specific antibodies targeting Flag (Flag-OTUB2, HA-KDM1A) at 4°C for 2 h and then protein A/G beads (40 µL) was added to each immunoprecipitation mixture at 4°C overnight. The beads were separated and washed by using cold phosphate-buffered saline, and then subjected to western blotting analysis.

For deubiquitination assay, polyUb was purified by IP using anti-KDM1A antibody (1 μg, Boster, Catalog No. M00532; Beijing, China) from cells transfected with OTUB2 shRNA after treated with MG-132. Thereafter, the poly-ubiquitination levels of KDM1A and protein levels of KDM1A were examined by anti-Ub antibody (abcam, Catalog No. Ab7254; 1:3000) and anti-KDM1A antibody (Affinity, Catalog No. DF6290; 1:2000), respectively.

### Statistical Analysis

Student’s t test and one-way ANOVA were used to analysis the difference among groups. Graphpad 8.0 for data analysis. GC patient survival curves were obtained from Kaplan-Meier plotter database. OTUB2 expression in GC tissues was extracted from TCGA database using GEPIA website. *P* < 0.05 was considered significantly.

## Results

### OTUB2 Is Overexpressed in GC Tissues and Cells and Is Preferentially Connected With Poor Prognosis of GC Patients

In order to determine whether the expression of OTUB2 is dysregulated in GC, we extracted the data from The Cancer Genome Atlas (TCGA) database and analyzed by the UALCAN website (http://ualcan.path.uab.edu/index.html). It was shown that OTUB2 was frequently upregulated in gastric tumor tissues compared with the normal (**Figure 1A**). The expression of OTUB2 was further explored in 140 pairs of GC tissues and corresponding normal tissues. As presented in **Figure 1B**, obviously higher OTUB2 expression was observed in GC tissues than that in adjacent tissues. Furthermore, the ratio of OTUB2 high expression to low expression in cancer tissues was significantly higher than that in adjacent tissues (**Figures 1C, D**). Moreover, we extracted GC patient survival curves from Kaplan-Meier plotter database (https://kmplot.com/analysis/). The results showed that patients with overexpression of OTUB2 indicated a shorter overall survival, first progression [the time from progression-free survival to the beginning of tumor progression after treatment (24)] and post progression survival (the time from tumor progression to death after treatment) compared with the patients with low expression of OTUB2 (**Figure 1E**). Further analysis showed that OTUB2 overexpression showed no significant association with age, gender, tumor size but was closely corrected with TNM stage, tumor differentiation, distal metastasis, and lymphatic metastasis (**Table 1**). Additionally, the OTUB2 protein expression in GC cell lines and GES-1 cells was further measured by Western blot. The results showed that OTUB2 expression was highly expressed in GC cells in comparison to the GES-1 cells (**Figure 2A**). These findings suggest that overexpression of OTUB2 is connected with poor prognosis of GC patients and may play a catalytic role in cancer progression.

**Table 1:** Correlations between OTUB2 expression and clinicopathologic characteristics in GC.

OTUB2 expression					
Characteristics	n = 140	Low (n = 57)	High (n = 83)	P value	X^2^
Gender				0.382	0.765
Male	65	29	36		
Female	75	28	47		
Age				0.562	0.337
<60	68	26	42		
≥60	72	31	41		
Tumor size(cm)				0.720	0.128
<3	86	34	52		
≥3	54	23	31		
Invasion				0.001	10.084
T0-T2	86	44	42		
T3-T4	54	13	41		
Lymphatic metastasis				<0.001	20.819
N0	89	49	40		
N1-4	51	8	43		
Tumor differentiation				0.003	9.050
Well/Moderately	82	42	40		
Poorly/undifferentiated	58	15	43		
Distal metastasis				0.028	4.803
M0	96	45	51		
M1	44	12	32		
TNM Stage				<0.001	18.575
0 & I & II	91	49	42		
III & IV	49	8	41		

**Figure 2:** Otubain 2 (OTUB2) promotes the maintenance of gastric cancer (GC) stem cell properties. **(A)** Relative protein expression levels of OTUB2 in GC cells (MKN-45, SGC-7901, SNU-1, HGC-27, and AGS) and gastric epithelial cells-1 (GES-1) were detected by Western blot. Actin served as internal control. **(B)** The protein levels of OTUB2, Nanog, ALDH, and Oct4 in GC cells were measured by Western blot after transfected with OTUB2 overexpression vector (MKN-45 and SGC-7901 cells) or shRNA targeting OTUB2 (HGC-27 and AGS cells). Actin served as internal control. **(C)** The effects of OTUB2 overexpression (MKN-45 and SGC-7901 cells) or knockdown (HGC-27 and AGS cells) on spheroid-forming ability were detected by sphere formation assay. **(D)** After cells were transfected with OTUB2 overexpression vector (MKN-45 and SGC-7901 cells) or shRNA targeting OTUB2 (HGC-27 and AGS cells), percentage of CD44 and CD133 double positive cells was detected by flow cytometry. Data was represented as mean ± SD. *P < 0.05, **P < 0.01, and ***P < 0.001.

### OTUB2 Promotes the Maintenance of GC Stem Cell Properties

To evaluate the effect of OTUB2 on GC stem cell properties, the HGC-27 and AGS cells were transfected with shRNAs targeting OTUB2 and MKN45 and SGC-7901 cells were transfected with OTUB2 overexpression plasmid. The efficiency of OTUB2 overexpression and interference was verified by Western blot (**Figure 2B**). Furthermore, OTUB2 overexpression obviously increased the protein expression levels of Nanog, ALDH, and Oct4 (CSC markers), while their protein levels were significantly decreased by OTUB2 silencing (**Figure 2B**). Spheroid formation assay indicated that upregulation of OTUB2 promoted the spheroid formation capacity of GC cells, whereas after downregulation of OTUB2, the spheroid formation was inhibited (**Figure 2C**). Flow cytometry analysis revealed that OTUB2 overexpression significantly increased CD44 and CD133 double (CSC markers) positive cells, whereas the CD44 and CD133 double positive cells were markedly decreased by knockdown of OTUB2 *via* shRNAs (**Figure 2D**). Overall, those data indicated that the high expression of OTUB2 is conducive to the maintenance of GC stem cell characteristics, while knockdown of OTUB2 has the opposite effect.

### OTUB2 Promotes the Proliferation, Invasion, and Migration of GC Cells

As CSCs facilitate the growth and metastasis of cancer cells, we further explored OTUB2-mediated effects on the proliferation, invasion, and migration of GC cells. As shown in **Figures 3A, B**, OTUB2 overexpression accelerated the growth of GC cells, while the viability and proliferation were suppressed in GC cells with OTUB2 silencing determined by MTT assay and EdU assay, respectively. Meanwhile, wound-healing and Transwell migration assays indicated that the ability of invasion and migration was enhanced by OTUB2 upregulation, but inhibited by OTUB2 downregulation (**Figures 3C, D**). Thus, the results suggested that OTUB2 contributes to the proliferation and metastasis of GC cells.

**Figure 3:** Otubain 2 (OTUB2) promotes the proliferation, invasion, and migration of gastric cancer (GC) cells. **(A)** Cell viability was detected in OTUB2-overexpressed (MKN-45 and SGC-7901 cells) or downregulated GC cells (HGC-27 and AGS cells). **(B)** Proliferating OTUB2-overexpressed (MKN-45 and SGC-7901 cells) or downregulated GC cells (HGC-27 and AGS cells) were labeled with EdU (red); cell nuclei were stained with DAPI (blue). Wound healing assays **(C)** and Transwell assays **(D)** were used to determine the changes in migratory and invasive abilities of GC cells transfected with OTUB2 overexpression vector (MKN-45 and SGC-7901 cells) or shRNA targeting OTUB2 (HGC-27 and AGS cells). Data was represented as mean ± SD. *P < 0.05, **P < 0.01, and ***P < 0.001.

### OTUB2 Promotes Xenograft Tumor Growth *In Vivo*

To investigate the effect of OTUB2 on xenograft tumor growth *in vivo*, stable transfection of HGC-27 and SGC-7901 cells with sh-OTUB2 or OE-OTUB2 were injected into nude mice. OTUB2 knockdown inhibited tumor growth, tumor volume as well as tumor weight, while OTUB2 overexpression had the opposite effects (**Figure 4A**). IHC staining showed that after injection of cells with stable low expression of OTUB2, OTUB2 and Ki67 (cell proliferation marker) expression in tumor tissues was decreased, whereas their expression was increased by OTUB2 overexpression (**Figure 4B**). These results revealed that OTUB2 serves as a positive regulator of tumor growth *in vivo*.

**Figure 4:** Otubain 2 (OTUB2) promotes xenograft tumor growth *in vivo.* **(A)** The nude mice were injected with GC cells, which were transfected with OTUB2 overexpression vector (SGC-7901 cells) or sh-OTUB2 (HGC-27 cells), respectively. Tumor volumes were calculated after injection every 5 days, tumor weight was measured 35 days after injection. **(B)** The tumor sections were underimmumohistochemical staining using antibodies against OTUB2 or Ki-67. Data was represented as mean ± SD. **P < 0.01.

### OTUB2 Increases the Stability of KDM1A

As a deubiquitinating enzyme, OTUB2 often affects the stability of genes by regulating the ubiquitination level of genes, and further participates in the development of diseases. Next, we explored whether OTUB2 promotes the maintenance of GC stem cell properties by influencing the stability of downstream genes in GC. Western blot analysis indicated that KDM1A protein level was significantly increased in OTUB2-overexpressed cells, whereas KDM1A expression was obviously decreased after OTUB2 inhibition (**Figure 5A**). We co-expressed Flag-OTUB2 and HA-KDM1A in 293T cells. Co-immunoprecipitation assay showed that when OTUB2 was immunoprecipitated, KDM1A was also pulled down. In turn, when KDM1A was immunoprecipitated, OTUB2 expression was also discovered (**Figure 5B**). Stable transfection of HGC-27 and MKN45 cells were treat with or without protease inhibitor MG132. The results showed that when protein degradation was inhibited, the ubiquitination of KDM1A was increased in OTUB2-downregulated cells compared with that in the normal cells, indicating that the increase in the ubiquitination level of KDM1A is due to the OTUB2 inhibition (**Figure 5C**). Furthermore, the stable transfection of HGC-27 and MKN45 cells were treated with or without cycloheximide (CHX, protein synthesis inhibitor). As presented in **Figure 5D**, in the presence of CHX, protein expression of KDM1A in OTUB2 overexpressed cells was higher than that in the control group at the same time point, while OTUB2 knockdown had the opposite effect, indicating that OTUB2 overexpression decreased the ubiquitination of KDM1A. Taken together, the results indicated that the effect of OTUB2 on KDM1A expression was achieved by regulating its ubiquitination.

**Figure 5:** Otubain 2 (OTUB2) increases the stability of KDM1A. **(A)** Relative protein levels of KDM1A in GC cells transfected with OTUB2 overexpression plasmids (MKN-45 and SGC-7901 cells) or shRNA targeting OTUB2 (HGC-27 and AGS cells). Actin served as internal control. **(B)** co-immunoprecipitation was conducted with anti-Flag (Flag-OTUB2) or anti-HA (HA-KDM1A) antibody and was analyzed by western blotting in 293T cells. **(C)** after transfected with shOTUB2, cells were treated with or without MG132. The ubiquitination level of KDM1A in MKN-45 and HGC-27 cells was measured by Western blot. Actin served as internal control. **(D)** After transfected with OTUB2 overexpression plasmids (MKN-45 cells) or shOTUB2, cells were treated with or without cycloheximide (CHX) for 0, 1, 2, 4, and 8 h, respectively. The protein expression levels of KDM1A were assessed by Western blot. Actin was used as internal control. Data was represented as mean ± SD. *P < 0.05, **P < 0.01, and ***P < 0.001.

### OTUB2 Promotes GC Stem Cell Properties Through Regulating KDM1A Expression

To explore whether KDM1A mediates the regulation of OTUB2 on the properties of GC stem cells, the correlation of OTUB2, KDM1A, and CD44 expression in GC tissues was first analyzed. IHC staining indicated that KDM1A and CD44 were highly expressed in tumor tissues with high expression of OTUB2 (**Figure 6A**). In contrast, low expression of KDM1A and CD44 was observed in tumor tissues with low expression of OTUB2 (**Figure 6A**). Correlation analysis showed that OTUB2 and KDM1A, OTUB2 and CD44, and KDM1A and CD44 all showed a significant positive regulatory relationship in GC tissues (**Figure 6B**). The regulatory relationship between OTUB2 and KDM1A was also verified in the tumor tissues of mice. The results showed that KDM1A expression in tumor tissues was increased by OTUB2 overexpression, but decreased by OTUB2 knockdown (**Figure 6C**). In addition, we inhibited the expression of KDM1A in OTUB2-overexpressed cells and found that inhibition of KDM1A reversed the promotion effects of OTUB2 overexpression on cell proliferation, migration, and invasion (**Figures 7A–D**). Meanwhile, we also enhanced KDM1A expression in OTUB2-downregulated cells. The results indicated that OTUB2 knockdown significantly decreased GC cell proliferation, migration, and invasion, which were inversed by KDM1A overexpression (**Figures 7A–D**). Additionally, the protein expression of KDM1A, Nanog, ALDH, and Oct4 was significantly increased by OTUB2 overexpression, while this increase was restored by KDM1A silencing (**Figure 7E**). Conversely, a significant decrease of KDM1A, Nanog, ALDH, and Oct4 expression was observed in OTUB2-downregulated cells, while KDM1A overexpression reversely increased their levels (**Figure 7E**). Taken together, those findings indicated that KDM1A mediated the regulation of OTUB2 on GC stem cells properties.

**Figure 6:** The expression of otubain 2 (OTUB2) and KDM1A in GC cells are positively correlated. **(A)** The expression of OTUB2, KDM1A, and CD44 was measured by immunohistochemistry in GC tissues collected from patients with GC. **(B)** The correlation between the expression of OTUB2, KDM1A, and CD44 in human tumor tissues was analyzed. **(C)** After OTUB2 was overexpressed (SGC-7901 cells) or downregulated (HGC-27 cells), the expression of KDM1A and CD44 was detected by immunohistochemistry in tumor tissues obtained from nude mice.

**Figure 7:** OTUB2 promotes GC stem cell properties through regulating KDM1A expression. **(B)** After MKN-45 cells were co-transfected with OTUB2 overexpression plasmids/NC and shKDM1A/Scr. The HGC-27 cells were co-transfected with shOTUB2/shNC and OV-KDM1A/vector, the cell viability was detected by MTT assay **(A)**; The spheroid-forming ability of GC cells were detected by sphere formation assay **(B)**. Wound healing assays **(C)** and Transwell assays **(D)** were used to determine the changes in migratory and invasive abilities of GC cells; Relative protein levels of KDM1A, Nanog, ALDH, and Oct4 IN GC cells were measured by Western blot **(E)**. Data was represented as mean ± SD. *P < 0.05, **P < 0.01, and ***P < 0.001. ^#^ *P* < 0.05, ^##^ *P* < 0.01, and ^###^ *P* < 0.001.

## Discussion

CSCs are subtypes of tumor cells with different functions, including multidirectional differentiation, self-renewal ability, high tumorigenicity, and chemotherapy resistance (25). CSCs have been successfully identified in various cancers, including GC (26), pancreatic cancer (27), and breast cancer (28). Currently, many treatments for CSCs have been proposed (29, 30). Researchers have isolated CSCs from many types of cancer, including GC (31). Studies have found that there is a considerable part of CD44 (+) cell subpopulations in GC cells, and these cells could form spherical colonies when cultured in serum-free medium (32). Additionally, CD44 (+) cells were tumorigenic *in vivo* and showed higher resistance to chemotherapy-induced or radiation-induced cell death (32). These studies suggest that CSCs have strong tumor initiation ability *in vivo* and may be an important target for GC therapy.

OTUB2 expression is dysregulated and plays a pro-carcinogenic role in a variety of cancers (8). However, whether OTUB2 affects the development of GC has not been reported. Present study found that OTUB2 was highly expressed in GC and was connected with the poor prognosis of GC patients, suggesting that OTUB2 may play a role in promoting GC progression. Many genes have been reported to regulate the maintenance of CSC properties in cancer progression. For example, CBX7 was significantly overexpressed in sphere cells from GC cells, and its overexpression increased the expression of stem cell markers CD44, CD24, and Oct-4 (26). Wang et al. (33) examined the expression of B cell-specific Moloney murine leukemia virus integration site 1 (Bmi-1) in microspheres and found that the expression of Bmi-1 and stem cell markers Oct-4, Sox2, Nanog, CD44, and CD133 was significantly increased in spheroid cells formed by SGC-7901 and MKN45 cells. However, whether OTUB2 regulates the maintenance of the stemness phenotype of GC cells is not yet known. We proved that OTUB2 induced stem cell properties of GC cells. The acquisition of cancer cell stemness enables epithelial cells to transform into a mesenchymal phenotype, which enhances cancer cell migration, invasion and resistance to apoptosis (34). We demonstrated that OTUB2 promoted the proliferation, migration and invasion of GC cells as well as the tumorigenicity of GC cells *in vivo*, indicating an important positive regulatory role of OTUB2 in GC progression. In view of the maintenance effect of OTUB2 on the stemness of GC cells, the promotion effect of OTUB2 on the cell function may be achieved by regulating the stemness of GC cells.

We next explored the potential molecular mechanism of OTUB2 regulating the stemness of GC cells. As a deubiquitinating enzyme, OTUB2 enhances gene stability by regulating the deubiquitination of downstream targets, including U2 small nuclear RNA auxiliary factor 2 (U2AF2) and Gli2 (6, 35). We demonstrated that OTUB2 increased KDM1A expression through deubiquitination. KDM1A is the first identified demethylase that can interact with a variety of protein complexes, transcription factors, receptors, etc. (36). It has been reported that KDM1A promoted cancer progression by removing methyl groups from the methylated histones H3 lysine 4 (H3K4) and H3 lysine 9 (H3K9) (37). KDM1A was overexpressed in various malignant tumors, including cervical cancer (38), esophageal cancer (39), ovarian cancer (40), and GC (41). The elevated KDM1A level was also related to tumor stage, histological grade, and lymph node metastasis (42). Additionally, KDM1A is a regulator of embryonic stem cells and can affect the self-renewal and differentiation of human embryonic stem cells (43). Given that the regulatory effect of KDM1A on embryonic stem cells, KDM1A may also affect the stemness of cancer cell.

Previous studies also proved this possibility that KDM1A was over-expressed in glioblastoma stem cells and its suppression reduced the self-renewal potential and viability of glioblastoma stem cells and at the same time induced cell apoptosis and differentiation (44). Herein, our results also proved that OTUB2 promoted the maintenance of GCSC properties through up-regulating KDM1A expression. Furthermore, Sareddy et al. (44) indicated that the activation of the unfolded protein response (UPR) pathway induced by KDM1A inhibitors reduced stem cells and induced differentiation and apoptosis in glioma stem cells. In addition, targeted inhibition of KDM1A eliminate sorafenib-resistant stem-like cells in hepatocellular carcinoma through blocking the Wnt/β-catenin signaling pathway (45). These findings indicated that KDM1A may participate in the regulation of CSC characteristics through multiple pathways. Moreover, it is worth noting that OTUB2, as a deubiquitinase, not only affects the stability of KDMIA, but also affects the stability of other proteins, such as YAP (11), Gli2 (35), which have been reported to promote GC progression (46, 47). Those findings indicate that OTUB2 can not only participate in the development of GC through KDMIA, but may also by regulating the expression of other proteins, such as YAP and Gli2. This also indicates the importance of OTUB2 in GC progression and its multi-pathway participation in the development of GC. Thus, OTUB2 inhibiton in GC tissues and cells may be a potential treatment for GC. Additionally, we noticed that there was a basal expression of OTUB2 in GC tissues and cells, indicating that OTUB2 inhibition may have side effects on normal tissues. However, our results combined with database (https://www.proteinatlas.org/) analysis showed that OTUB2 expression was quite low in normal tissues. Therefore, therapies for targeted inhibition of OTUB2 may have little side effects on normal cells, or even not enough to affect their function. This also suggests that OTUB2 may be a promising therapeutic target. As we demonstrated that OTUB2 overexpression promoted GC proliferation and inhibited apoptosis, indicating that the basic expression of OTUB2 in normal cells may be related to normal cell functions, such as proliferation and apoptosis. Moreover, OTUB2 protein expression was observed in human gastric epithelium GES-1 cells, this suggests that human gastric epithelium GES-1 cells may be one of types expressing OTUB2. However, whether there are other gastric cells expressing OTUB2 needs further exploration. For the functions and locations of OTUB2 in non-cancerous tissues and cells, another well-designed study will be performed in the future. Collectively, we first investigated the function of OTUB2 in GC progression and the underlying molecular mechanism. We found that OTUB2 positively regulated stem cell-like characteristics of GC cells and further enhanced the proliferation, invasion, and migration of GC cells. This was achieved by increasing the stability of KDM1A through deubiquitination. Our findings provide strong evidence for OTUB2 may be a potential target for the treatment of GC.

## Data Availability Statement

The original contributions presented in the study are included in the article/supplementary material. Further inquiries can be directed to the corresponding author.

## Ethics Statement 

All procedures performed in studies involving human participants were in accordance with the standards upheld by the Ethics Committee of The First Hospital of Jilin University and with those of the 1964 Helsinki Declaration and its later amendments for ethical research involving human subjects. The patients/participants provided their written informed consent to participate in this study. All animal experiments were approved by the Ethics Committee of The First Hospital of Jilin University for the use of animals and conducted in accordance with the National Institutes of Health Laboratory Animal Care and Use Guidelines.

## Author Contributions

GL and WG designed the study, supervised the data collection. JQ analyzed the data and interpreted the data. ZL prepare the manuscript for publication and reviewed the draft of the manuscript. All authors contributed to the article and approved the submitted version.

## Conflict of Interest

The authors declare that the research was conducted in the absence of any commercial or financial relationships that could be construed as a potential conflict of interest.

## Publisher’s Note

All claims expressed in this article are solely those of the authors and do not necessarily represent those of their affiliated organizations, or those of the publisher, the editors and the reviewers. Any product that may be evaluated in this article, or claim that may be made by its manufacturer, is not guaranteed or endorsed by the publisher.
